The article "Analysis of Prognostic Factors and Construction of Prognostic Models for Invasive Micropapillary Carcinoma of the Breast" was published in 2022. Journal: Comput Math Methods Med.

# Analysis of Prognostic Factors and Construction of Prognostic Models for Invasive Micropapillary Carcinoma of the Breast

**DOI:** 10.1155/2022/1072218

**Published:** 2022-10-26

**Authors:** Xinli Wang, Yan Xue

**Affiliations:** Xi'an International Medical Center Hospital, Xi'an, Shaanxi Province 710100, China

## Abstract

**Objective:**

To compare and analyze the clinical characteristics of invasive micropapillary carcinoma (IMPC) of the breast (IMPC-B) and invasive ductal carcinoma (IDC) of the breast (IDC-B) and establish a prognostic model of IMPC-B.

**Methods:**

We retrospectively analyzed data for patients diagnosed with breast cancer in the Surveillance, Epidemiology, and End Results (SEER) database between 2010 and 2018 and screened 581 patients with IMPC and 1325 patients with IDC. We compared age, race, laterality, tumor site, histological grade, type of surgery, radiation, chemotherapy, whether the first primary tumor, T stage, N stage, M stage, and molecular type between IMPC-B and IDC-B and draw survival curves of IMPC-B and IDC-B. The relationship between clinical factors and prognosis was investigated by univariate analysis using the Log-rank test and multivariate analysis of the Cox proportional hazards regression model. A risk scoring model was constructed based on independent risk factors to distinguish high-risk and low-risk patients; in addition, a nomogram was created to predict patient survival.

**Results:**

There were differences between the two groups in the age of onset, race, tumor site, histological grade, type of surgery, N stage, and molecular type (*p* < 0.05). Overall survival was decreased in IMPC-B compared with IDC-B (*p* < 0.05). The prognosis of IMPC-B was significantly correlated with histological grade, whether the first primary tumor, type of surgery, radiotherapy, chemotherapy, T stage, and N stage. Based on the relationship between the above factors and overall survival prognosis, the risk score model we constructed can effectively distinguish high-risk and low-risk patients (*p* < 0.05). The established nomogram had better performance in predicting survival in patients with IMPC-B (C − index = 0.78).

**Conclusion:**

IMPC-B has a worse prognosis than IDC-B, with earlier age of onset, higher histological grade, and later N stage, and luminal breast cancer is the main type. The nomogram can well predict the prognosis of patients with IMPC-B, which has a high clinical reference value and provides a scientific basis for clinical treatment.

## 1. Introduction

Invasive micropapillary carcinoma is a special histological subtype of breast cancer, accounting for 2% to 8% of breast cancers [1]. So far, IMPCs have been reported in multiple organs, including the lung, bladder, colon, and pancreas. Pure IMPC is rare and often coexists with other histological types. Morphologically, tumor cells of IMPC have papillary or glandular-like structures, no fibrovascular bundles in the center of cell clusters, cell membrane antigen (EMA) staining shows polarity reversal, tight junctions between tumor cells, and cell clusters are mostly unconnected to the stroma. A small number of tumor cell clusters were in contact with the stroma, and the contact side was rich in E-cadherin, rich in motor fibers, mitochondria, etc. The interstitium contains a large number of new capillaries, lymphatic vessels, and myofibroblasts. IMPC is aggressive in groups [2, 3]. The unique clustered growth pattern and aggressive biological behavior of IMPC make it more invasive and prone to vascular invasion and lymph node metastasis [4, 5]. Previous studies have shown that even if the tumor is less than 2 cm, and the proportion of tumor tissue is less than 25%, the number of lymphatic invasions, lymph node metastasis, and lymph node metastasis of IMPC is significantly higher than that of invasive ductal carcinoma. Therefore, they propose a pathological diagnostic standard for diagnosing and indicating the proportion of invasive papillary carcinoma as long as there are invasive papillary carcinoma components in the cancer tissue [6]. However, there is no unified conclusion on its clinicopathological characteristics and prognostic factors. How comprehensively considering the risk factors of IMPC-B patients and predicting the prognosis is of great significance to improve the survival of IMPC-B patients.

The article "Analysis of Prognostic Factors and Construction of Prognostic Models for Invasive Micropapillary Carcinoma of the Breast" was published in 2022. Journal: Comput Math Methods Med.

Surveillance, Epidemiology, and End Results (SEER) is a repository of survival statistics from community-based cancer registries covering about 28% of the US population [7, 8]. The purpose of this study was to compare and analyze the data of IMPC-B and IDC-B patients, analyze the clinical factors affecting IMPC-B, and distinguish between high-risk and low-risk patients. A nomogram model for predicting the overall survival (OS) rate of patients was constructed to provide a basis for individualized treatment of patients.

## 2. Materials and Methods

### 2.1. Materials

The data of IMPC-B patients and IDC-B patients in the SEER database from 2010 to 2018 were extracted by SEER^∗^Stat software (version 8.3.6.1), 581 IMPC-B and 1325 IDC-B patients were included. Inclusion criteria: (1) patients with pathologically diagnosed breast cancer; (2) pathologically classified as IMPC or IDC; (3) complete clinicopathological characteristics and follow-up data. Exclusion criteria: (1) Important information such as differentiation degree, tumor stage, molecular typing, and treatment was missing; (2) follow-up information was incomplete.

The article "Analysis of Prognostic Factors and Construction of Prognostic Models for Invasive Micropapillary Carcinoma of the Breast" was published in 2022. Journal: Comput Math Methods Med.

### 2.2. Ethical Review

We obtained signed authorization and permission to access and use data from the SEER database and adhered to protocols throughout to protect patient privacy. The Ethics Committee of Xi'an International Medical Center Hospital approved the ethical requirements for this study. This study was conducted by the revised Declaration of Helsinki.

### 2.3. Statistical Analysis

Baseline characteristics of IMPC-B and IDC-B were compared using the *χ*2 test and Fisher's exact test, and Kaplan-Meier was used to draw survival curves of IMPC-B and IDC-B. The relationship between clinical factors and prognosis was investigated by univariate analysis using the Log-rank test, and variables that may be related to prognosis were screened out. These screened variables were then subjected to multivariate analysis of the Cox proportional hazards regression model to determine the independent risk factors affecting the prognosis of IMPC-B. MedCalc software was used to calculate the Youden index, and the median of the Youden index of all patients was used as the cutoff value. Those higher than or equal to the median were considered high risk, and those lower than the median were considered low risk. Kaplan-Meier was used to draw survival curves of the high-risk group and the low-risk group, and a risk scoring model was constructed. Nomograms were performed using R software (4.0.3). The reliability of the model was verified by the calibration curve and receiver operating characteristic curve (ROC). *P* < 0.05 was considered a statistically significant difference.

## 3. Results

### 3.1. Comparison of Clinicopathological Characteristics and Survival between IMPC-B and IDC-B Patients

IMPC-B and IDC-B patients were statistically significant in terms of age, race, tumor site, histological grade, type of surgery, chemotherapy, N stage, and molecular type (*P* < 0.05, Table 1). Compared with IDC-B, IMPC-B patients have a younger age of onset, higher proportion of central and upper-inner quadrant tumors, higher histological grade, higher lymph node metastasis rate, and a higher proportion of HER2-positive breast cancer and require postoperative adjuvant chemotherapy. The Kaplan-Meier survival curve showed that the survival prognosis of IMPC-B patients was significantly worse than that of IDC-B (*P* < 0.05, Figure 1).

### 3.2. Analysis of Prognostic Factors of IMPC-B

The results of analysis using univariate and Cox proportional hazards regression model showed that histological grade, type of surgery, radiotherapy, chemotherapy, and whether the first primary tumor, T stage, and N stage were independent risk factors for OS prognosis in IMPC-B patients (*P* < 0.05, Table 2).

The article "Analysis of Prognostic Factors and Construction of Prognostic Models for Invasive Micropapillary Carcinoma of the Breast" was published in 2022. Journal: Comput Math Methods Med.

### 3.3. Construction and Verification of Risk Scoring Model Based on Independent Risk Factors

Risk scores for the histological grade, type of surgery, radiotherapy, chemotherapy, and whether the first primary tumor, T stage, and N stage were calculated. Patients were divided into high/low-risk groups according to the median of the Youden index. The distributions of risk factor-based risk scores, OS status, and risk factor expression profiles were shown in Figure 2(a). Risk factors were more expressed in patients in the high-risk group. Kaplan-Meier curve analysis clearly showed that the high-risk group had a worse prognosis than the low-risk group (*χ*2 = 33.013, *p* = 0.001) (Figure 2(b)).

### 3.4. Creating a Nomogram Based on Clinical Risk Factors

We integrated histological grade, type of surgery, radiotherapy, chemotherapy, whether first primary tumor, T stage, and N stage to develop an efficient quantitative method for predicting OS, which was a nomogram. We used the nomogram to predict 1-, 3-, and 5-year survival in patients with IMPC-B (Figure 3). We plotted the 1-, 3-, and 5-year ROC curves and calculated the corresponding AUCs (Figure 4). The 1-, 3-, and 5-year AUCs were 0.940, 0.943, and 0.943, respectively. We then plotted calibration plots to verify the consistency between the actual and ideal values of the model after verifying its discrimination ability. As shown in Figure 5, the calibration plots for 1-, 3-, and 5-year OS probabilities for the model are very close to the standard lines. Internal validation using bootstrap with 1000 resamplings revealed that the nomogram performed well for discrimination, with a C-index of 0.78. Therefore, the prediction performance of the risk prediction model was good. Finally, DCA curves were used to illustrate the clinical effectiveness of the nomogram, and the results showed that the model to predict the 1-, 3-, and 5-year OS probabilities was good (Figure 6).

## 4. Discussion

Due to the highly heterogeneous nature of breast cancer, there are significant individual differences between breast cancer patients [9], even patients of breast cancer with the same histological type, TNM stage, and even hormone receptor status, using the same standard treatment regimen recommended by the clinical guidelines, the efficacy and prognosis are often very different [10], so it is extremely important to individualize the treatment of breast cancer patients. The premise of individualized treatment is to accurately predict the biological behavior of breast cancer. Therefore, the development of a highly reliable and repeatable prognostic prediction system that provides a quantitative prognostic index is crucial for guiding individualized comprehensive treatment. Nomograms can make an individualized prediction of survival at a specific time point. As a new prediction model, compared with traditional prediction methods, it has higher accuracy, wider adaptability, and is easy to generalize [11]. IMPC is a special type of breast cancer with a low incidence of overall breast cancer. Most studies have shown that IMPC-B is highly invasive and has a poor prognosis [12, 13]. Due to its high invasiveness and high mortality, its pathogenesis mechanism and prognostic factors deserve further study.

The article "Analysis of Prognostic Factors and Construction of Prognostic Models for Invasive Micropapillary Carcinoma of the Breast" was published in 2022. Journal: Comput Math Methods Med.

This study analyzed the clinicopathological characteristics of IMPC-B and compared them with IDC-B to better understand the biological characteristics of IMPC-B. The incidence of IMPC-B is high in white people, mostly in the upper-outer quadrant of the breast, and more common in HR+/HER2-. Compared with IDC-B, the age of onset of IMPC-B patients was younger, and the proportion of tumors in the central region and upper-inner quadrant increased. The proportion of IMPC-B cases with histological grade III accounted for 33.2%, which was significantly higher than that of IDC-B (15%); the rate of lymph node metastasis was higher than IDC-B (43.5% vs. 30.9%), which is consistent with previous studies [6, 14]; IMPC-B is more common in HR+/HER2-, which is consistent with previous reports [15], and this study found that HER2-positive rate of IMPC-B patients was higher than that of IDC-B, 19.6% vs. 9.0%, and HR+/HER2+ were more common. The rate of postoperative adjuvant chemotherapy in IMPC-B was higher than that in IDC-B, which was associated with a poorer prognosis in IMPC-B. The Kaplan-Meier survival curve of this study verified that the survival prognosis of IMPC-B patients was significantly worse than that of IDC-B. Multivariate analysis showed that histological grade, type of surgery, radiotherapy, chemotherapy, and whether the first primary tumor, T stage, and N stage were independent risk factors for IMPC-B. The prognostic risk model created based on the above factors can effectively distinguish between high- and low-risk patients, and the survival time of high-risk patients was significantly shorter than that of low-risk patients. Risk scoring models can guide clinical treatment, to a certain extent, avoid overtreatment of low-risk patients, and adopt more aggressive treatment strategies for high-risk patients. This study constructed a nomogram prediction model, AUC = 0.779, and C − index = 0.78, and the calibration plots and DCA curves showed that the nomogram has a good prognosis prediction ability.

The article "Analysis of Prognostic Factors and Construction of Prognostic Models for Invasive Micropapillary Carcinoma of the Breast" was published in 2022. Journal: Comput Math Methods Med.

In terms of biological behavior, IMPC-B has the characteristics of high lymphatic invasion, high lymph node metastasis, high recurrence, and high distant metastasis even if the tumor is less than 2 cm, or the IMPC component in mixed breast cancer accounts for less than 25%. Researchers have proposed that it is not the size of the tumor or the number of IMPC components that correlates with tumor aggressive behavior, but the presence of IMPC components [3, 6]. Therefore, regardless of the proportion of IMPCs in tumors, clinicians should pay attention. This study found that the proportion of breast-conserving surgery of IMPC was significantly higher than that of IDC-B patients, which may be related to small tumors and incomplete assessment before surgery, suggesting the importance of comprehensive and accurate preoperative assessment. Multifocal punctures and aggressive surgical approaches may benefit patients.

## 5. Conclusion

This study established a prediction model based on the data of IMPC-B patients in the SEER database and established independent risk factors for the prognosis of IMPC-B patients, and predictive models can accurately and effectively predict the prognosis of patients with IMPC-B, which can help individualized management of IMPC-B patients.

## Figures and Tables

**Figure 1:** K-M curves of IDPC-B and IDC-B.

**Figure 2:** Risk scoring model. (a) Risk score distribution, survival status, and heat map of risk factor markers; (b) K-M curve of the high/low-risk group.

**Figure 3:** Nomogram to predict 1/3/5-year overall survival of IMPC-B patients.

**Figure 4:** ROC curve for predicting 1/3/5-year overall survival of IMPC-B patients with the nomogram.

**Figure 5:** Calibration curve of the nomogram for 1-, 3-, and 5-year OS probability(C − index = 0.78).

**Figure 6:** Decision curve analysis curves. Decision curve for 1-, 3-, and 5-year OS probability.

**Table 1:** Clinical characteristics and comparison of IMPC-B and IDC-B patients.

Factors	IMPC *n* = 581	IDC *n* = 1325	*χ*2	*P* value
Age (*y*)			1141.009	0.001
<35	13 (2.2%)	9 (0.7%)		
35-59	228 (39.2%)	502 (37.9%)		
≥60	340 (58.5%)	814 (61.4%)		
Race			15.169	0.001
Black	75 (12.9%)	115 (8.7)		
White	438 (75.4)	1100 (83.0)		
Other	68 (11.7)	110 (8.3)		
Laterality			0.472	0.492
Left	291 (50.1)	641 (48.4)		
Right	290 (49.9)	684 (51.6)		
Tumor site			20.100	0.001
The central portion of breast	40 (6.9)	76 (5.7)		
Upper-inner quadrant	87 (15.0)	174 (13.1)		
Lower-inner quadrant	58 (10.0)	68 (5.1)		
Upper-outer quadrant	203 (34.9)	537 (40.5)		
Lower-outer quadrant	45 (7.7)	108 (8.2)		
Overlapping lesion of breast	148 (25.5)	362 (27.3)		
Histological grade			125.508	0.001
I	39 (6.7)	307 (23.2)		
II	349 (60.1)	819 (61.8)		
III	193 (33.2)	199 (15.0)		
Type of surgery			567.821	0.001
Partial mastectomy	316 (54.4)	148 (11.2)		
Total mastectomy	127 (21.9)	1007 (76.0)		
Radical mastectomy	119 (20.5)	170 (12.8)		
No	19 (3.3)	0 (0)		
Radiation			2.324	0.127
Yes	345 (59.4)	737 (55.6)		
No	236 (40.6)	588 (44.4)		
Chemotherapy			60.688	0.001
Yes	277 (47.7)	387 (29.2)		
No	304 (52.3)	938 (70.8)		
Whether the first primary tumor			0.674	0.412
Yes	492 (84.7)	1102 (83.2)		
No	89 (15.3)	223 (16.8)		
T stage			5.017	0.171
T1	337 (58.0)	818 (61.7)		
T2	182 (31.3)	401 (30.3)		
T3	44 (7.6)	81 (6.1)		
T4	18 (3.1)	25 (1.9)		
N stage			47.546	0.001
N0	328 (56.5)	916 (69.1)		
N1	163 (28.1)	321 (24.2)		
N2	49 (8.4)	55 (4.2)		
N3	41 (7.1)	33 (2.5)		
M stage			0.026	0.872
M0	564 (97.1)	1288 (97.2)		
M1	17 (2.9)	37 (2.8)		
Molecular subtype			47.057	0.001
HR+/HER2-	449 (77.3)	1180 (89.1)		
HR+/HER2+	92 (15.8)	101 (7.6)		
HR-/HER2+	22 (3.8)	18 (1.4)		
HR-/HER2-	18 (3.1)	26 (2.0)		

The article "Analysis of Prognostic Factors and Construction of Prognostic Models for Invasive Micropapillary Carcinoma of the Breast" was published in 2022. Journal: Comput Math Methods Med.

**Table 2:** Univariate and multivariate analyses of breast IMPC patients.

Factors	Univariate analysis		Multivariate analysis		
	*χ*2	*P* value	Risk ratio (HR)	95% confidence interval	*P* value
Age (*y*)	7.520	0.023			0.241
<35			1		
35-59			4096.629	0.000 − 2.259*E*48	0.874
≥60			6574.659	0.000 − 3.624*E*48	0.867
Race	5.664	0.059	—		—
Black					
White					
Other					
Laterality	1.039	0.308	—		—
Left					
Right					
Tumor site	3.743	0.587	—		—
The central portion of breast					
Upper-inner quadrant					
Lower-inner quadrant					
Upper-outer quadrant					
Lower-outer quadrant					
Overlapping lesion of breast					
Histological grade	10.414	0.015			0.004
I			1		
II			0.678	0.227 − 2.024	0.487
III			1.875	0.600 − 5.859	0.280
Type of surgery	51.392	0.001			0.030
Partial mastectomy			1		
Total mastectomy			0.736	0.328 − 1.651	0.458
Radical mastectomy			0.919	0.381 − 2.213	0.850
NO			4.405	1.287 − 15.082	0.018
Radiation	18.764	0.001	0.402	0.208 − 0.780	0.007
Yes					
No					
Chemotherapy	6.170	0.013	0.292	0.148 − 0.574	0.001
Yes					
No					
Whether the first primary tumor	10.164	0.006	0.333	0.173 − 0.642	0.001
Yes					
No					
T stage	38.963	0.001			0.011
T1			1		
T2			1.438	0.733 − 2.823	0.291
T3			3.139	1.082 − 9.106	0.035
T4			9.036	2.303 − 35.450	0.002
N stage	13.360	0.004			0.035
N0			1		
N1			0.902	0.418 − 1.945	0.793
N2			2.507	0.847 − 7.425	0.097
N3			3.847	1.265 − 11.703	0.018
M stage	9.612	0.002	2.250	0.825 − 6.137	0.113
M0					
M1					
Molecular subtype	2.284	0.516	—		—
HR+/HER2-					
HR+/HER2+					
HR-/HER2+					
HR-/HER2-					

## Data Availability

All supporting data are included within the main article.

The article "Analysis of Prognostic Factors and Construction of Prognostic Models for Invasive Micropapillary Carcinoma of the Breast" was published in 2022. Journal: Comput Math Methods Med.

## References

[1] Guan X., Xu G., Shi A. (2020). Comparison of clinicopathological characteristics and prognosis among patients with pure invasive ductal carcinoma, invasive ductal carcinoma coexisted with invasive micropapillary carcinoma, and invasive ductal carcinoma coexisted with ductal carcinoma in situ: a retrospective cohort study. *Medicine(Baltimore).*.

[2] Yang Y. L., Liu B. B., Zhang X., Fu L. (2016). Invasive micropapillary carcinoma of the breast: an update. *Archives of Pathology & Laboratory Medicine*.

[3] Fu L., Ikuo M., Fu X. Y., Liu T. H., Shinichi T. (2004). Relationship between biologic behavior and morphologic features of invasive micropapillary carcinoma of the breast. *Zhonghua Bing Li Xue Za Zhi*.

[4] Ye F., Yu P., Li N. (2020). Prognosis of invasive micropapillary carcinoma compared with invasive ductal carcinoma in breast: a meta-analysis of PSM studies. *Breast*.

[5] Jenkins S., Kachur M. E., Rechache K., Wells J. M., Lipkowitz S. (2021). Rare breast cancer subtypes. *Current Oncology Reports*.

[6] Guo X., Chen L., Lang R., Fan Y., Zhang X., Fu L. (2006). Invasive micropapillary carcinoma of the breast. *American Journal of Clinical Pathology*.

[7] Yang J., Li Y., Liu Q. (2020). Brief introduction of medical database and data mining technology in big data era. *Journal of Evidence-Based Medicine*.

[8] Wu W. T., Li Y. J., Feng A. Z. (2021). Data mining in clinical big data: the frequently used databases, steps, and methodological models. *Military Medical Research*.

[9] Simpson P. T., ReisFilho J. S., Lakhani S. R. (2010). Breast pathology: beyond morphology. *Seminars in Diagnostic Pathology*.

[10] Park Y. H., Lee S. J., Cho E. Y. (2011). Clinical relevance of TNM staging system according to breast cancer subtypes. *Annals of Oncology*.

[11] Balachandran V. P., Gonen M., Smith J. J., DeMatteo R. P. (2015). Nomograms in oncology: more than meets the eye. *The Lancet Oncology*.

[12] Han C. H., Yao W. G., He J., Gao Z.‑. B., Hu H.‑. J. (2020). MRI and the pathology of breast invasive micropapillary carcinoma. *Oncology Letters*.

[13] Li D., Zhong C., Cheng Y. (2019). A competing nomogram to predict survival outcomes in invasive micropapillary breast cancer. *Journal of Cancer*.

[14] Li W., Han Y., Wang C. (2018). Precise pathologic diagnosis and individualized treatment improve the outcomes of invasive micropapillary carcinoma of the breast: a 12-year prospective clinical study. *Modern Pathology*.

[15] Deman F., Punie K., Laenen A. (2020). Assessment of stromal tumor infiltrating lymphocytes and immunohistochemical features in invasive micropapillary breast carcinoma with long-term outcomes. *Breast Cancer Research and Treatment*.

